# Assessment of Myocardial Work of the Left Ventricle before and after PCI in Patients with Non-ST-Segment Elevation Acute Coronary Syndrome by Pressure-Strain Loop Technology

**DOI:** 10.1155/2022/8026689

**Published:** 2022-05-26

**Authors:** Fei Ren, Ting Xue, Ge Tang, Man Zhang, Jing Zhao, Yun'An Chen, Jixu Fan, Ming Yu, Jie Zhang

**Affiliations:** ^1^Department of Science and Education, The First Affiliated Hospital of Kangda College of Nanjing Medical University/The First People's Hospital of Lianyungang, Lianyungang 222002, China; ^2^Department of Heart Function Test, The First Affiliated Hospital of Kangda College of Nanjing Medical University/The First People's Hospital of Lianyungang, Lianyungang 222002, China; ^3^Department of Ultrasound, The Affiliated Lianyungang Hospital of Xuzhou Medical University, Lianyungang 222002, China

## Abstract

**Objectives:**

Noninvasive left ventricular pressure-strain loop (PSL) is a new method for quantitative evaluation of myocardial work, which is developed on the basis of speckle tracking echocardiography. It is necessary to fit the noninvasive left ventricular pressure and the strain by speckle tracking echocardiography to construct a pressure-strain loop. Compared with traditional left ventricular ejection fraction (LVEF) and global longitudinal strain (GLS), it has potential application value and is a useful supplement for clinical evaluation of left ventricular systolic function. We perform this study to evaluate the changes of myocardial function in patients with non-ST-segment elevation acute coronary syndrome (NSTE-ACS) before and after percutaneous coronary intervention (PCI) with noninvasive left ventricular pressure-strain loop (PSL).

**Methods:**

33 NSTE-ACS patients admitted to the Department of Cardiovascular Medicine of the Affiliated Lianyungang Hospital of Xuzhou Medical University who successfully underwent early PCI were included as the PCI group. At the same time, 30 healthy patients matched in age and sex were selected as the control group. All patients received routine echocardiography. The parameters such as GWI, GCW, GWW, and GWE were obtained by EchoPAC 203 software. The differences in the general clinical data and echocardiographic parameters between the two groups, including controls and patients 1 day before surgery and 1 month after surgery, were compared.

**Results:**

Compared with the control group, GWI, GCW, and GWI in the PCI group were decreased 1 day before surgery and 1 month after surgery, while GWW was increased, with statistical significance (*P* < 0.05). In the PCI group, compared with 1 day before surgery, GWI and GCW were all increased 1 month after surgery (*P* < 0.05), and GWW and GWE were not significantly different between the two groups (*P* > 0.05).

**Conclusion:**

The noninvasive left ventricular PSL technology can early and accurately evaluate the myocardial function impairment in NSTE-ACS patients and the recovery of myocardial function after PCI, providing a new noninvasive method for clinical postoperative myocardial function evaluation.

## 1. Introduction

Non-ST-segment elevation acute coronary syndrome (NSTE-ACS) is one of the main cardiovascular diseases, which seriously impairs humanity's life and health. In recent years, the incidence and fatality rate of NSTE-ACS gradually increased and tended to be younger. Percutaneous coronary intervention (PCI) restores the normal blood flow of the coronary artery through treatment of stenosis [1], effectively opens the coronary artery stenosis, restores myocardial perfusion, and timely improves the myocardial systolic function of patients. It is an effective treatment for NSTE-ACS. In recent years, the evaluation of left ventricular structure and function changes after PCI has always been a research hotspot. Echocardiography is an effective imaging method to evaluate left ventricular myocardial function after PCI due to its advantages of noninvasive, simple operation, economic, and strong operability.

Noninvasive left ventricular pressure-strain loop (PSL) is a new technology based on two-dimensional speckle-tracking echocardiography (2D-STE) in recent years. The myocardial work (MW) obtained by PSL provides a new parameter for quantitative evaluation of left ventricular systolic function from the perspective of myocardial mechanics. PSL technology simultaneously combines the global longitudinal strain (GLS) of 2D-STE and left ventricular pressure (replaced by brachial artery systolic and diastolic blood pressure measured by a noninvasive cuff sphygmomanometer) to overcome the influence of GLS load conditions [2]. A recent study showed that left ventricular PSL provides a unique method of quantifying MW, superior to conventional EF and GLS [3]. At present, there are more and more studies on the diagnosis and prognosis of coronary heart disease with PSL, but there are few studies on the myocardial work of NSTE-ACS patients after PCI. In this study, the changes of left ventricular cardiac function in NSTE-ACS patients before and after PCI were mainly investigated by PSL technology.

## 2. Materials and Methods

### 2.1. Study Population

This study is performed at a single heart center at the Affiliated Lianyungang Hospital of Xuzhou Medical University. From September 2020 to April 2021, 33 patients with the diagnosis NSTE-ACS [4] who underwent coronary angiography and initial PCI were enrolled in this study and were followed up for 1 month. There were 25 males and 8 females aged from 38 to 76 years, with an average of 62.09 ± 9.16 years. Blood pressure of all the patients should be kept within the normal range, regardless of whether the patient is hypertensive or not, as wide fluctuations in blood pressure can affect PSL results. A total of 48 vessels (stenosis ≥ 75% in diameter of the coronary artery) were detected in 33 patients, including 21 left anterior descending artery, 12 circumferential artery, and 15 right coronary artery. There were 22 cases of single-vessel coronary stenosis, 7 cases of two-vessel coronary stenosis, and 4 cases of three-vessel coronary stenosis. All patients underwent related echocardiography and brachial artery blood pressure measurement 1 day before surgery and 1 month after surgery. At the same time, 30 healthy subjects with matched age were selected as the control group, including 20 males and 10 females, aged from 43 to 71 years, with an average of 58.50 ± 6.70 years.

Inclusion criteria were as follows: patients with the clinical diagnosis of NSTE-ACS; coronary angiography showing at least one coronary artery stenosis ≥ 75%; and all subjects had LVEF ≥ 55% and no segmental wall motion abnormalities. Exclusion criteria were as follows: previous history of myocardial infarction; patients previously treated with PCI or CABG; patients with cardiomyopathy, valvular disease, and arrhythmia (atrial fibrillation, complete left bundle branch block, etc.); and patients without high quality of two-dimensional ultrasonic images.

All participating subjects signed written informed consent on the research, and the study was approved by the Ethics Committee of Lianyungang First People's Hospital.

### 2.2. Echocardiography

#### 2.2.1. Conventional Echocardiography

The conventional transthoracic echocardiography was performed using an available GE Vivid E95 ultrasound system (Vingmed Ultrasound, Horten, Norway) with an M5S 1.5~4.0 MHz transducer. All images were stored and analyzed on the EchoPAC 203 workstation (GE Healthcare). All procedures were performed by the same experienced sonographer according to the guidelines of the American Society of Echocardiography [5, 6]. None of the patients had chest pain at the time of echocardiography. Echocardiography was performed once in the control group during physical examination, and echocardiography was performed 1 day before surgery and 1 month after surgery in the PCI group.

Echocardiography was performed when patients were at rest in left decubitus position, and the electrocardiograph was connected synchronously. Systolic and diastolic blood pressures of the brachial artery were measured by a cuff sphygmomanometer before operating, and height and weight of patients were recorded. Left anteroposterior atrial diameter (LAD), left ventricular end systolic diameter (LVIDd), and left ventricular end diastolic diameter (LVIDs) were measured in the long-axial view of the left ventricle by conventional echocardiography. Left ventricular ejection fraction (LVEF) was measured according to the modified biplane Simpson method in the apical four-chamber view. The peak value (*E*) of mitral valve early diastolic flow velocity was obtained via pulsed-wave Doppler echocardiography. The average of the septal and lateral annulus mitral early diastolic (*e*′) tissue Doppler velocity and the *E*/*e*′ ratio were calculated. All data are averages of three measurements.

#### 2.2.2. Two-Dimensional Speckle-Tracking Echocardiography and Myocardial Work

The standard images we need to acquire include the dynamic images of the left ventricular apical four-chamber, three-chamber, and two-chamber view, with 3 consecutive cardiac cycles and frame rate > 40% of heart rate. All images were imported into EchoPAC 203 workstation in the original image format for postprocessing offline.

The opening and closing time of mitral and aortic valves was determined by the three-chamber view of the apex, and GLS was obtained by AFI. Subsequently, click on myocardial work to obtain PSL, global work index (GWI), global constructive work (GCW), global wasted work (GWW), and global work efficiency (GWE). GWI refers to the area of the left ventricular PSL and the sum of the work done by the myocardium from mitral valve closure to mitral valve opening. GCW is the work done by the myocardium during systolic shortening or isovolemic diastolic lengthening, which contributes to left ventricular ejection. In contrast, GWW is the work done by the myocardium during prolonged systole or shortened isovolemic diastolic phase, blocking left ventricular ejection. GWE is the percentage of GCW in the sum of GCW and GWW, reflecting the efficiency of mechanical energy to do work in the whole cardiac cycle. Apparently, this increased effort reduces the heart's ability to shoot blood, making the heart muscle less efficient at doing its work and ultimately leading to heart failure and even death.

### 2.3. Statistical Analysis

The data were analyzed using IBM SPSS Statistics version 22.0 (IBM SPSS Statistics for Windows, Armonk, NY). Continuous variables are expressed by their mean and standard deviation if normally distributed. Continuous data were compared using the Student *t* test or Kruskal-Wallis rank sum test between two groups. Comparison of continuous variables among more than two groups was analyzed by one-way analysis of variance or Kruskal-Wallis rank sum test. Categorical data are expressed in terms of frequencies and percentage and were compared with the *χ*^2^ test. Correlation between GLS and MW parameters of the left ventricle was analyzed by Pearson correlation analysis. Images of 10 patients were randomly selected from the two groups, and the inter- and intraobserver agreement of GWI, GCW, GWW, and GWE was assessed by intraclass correlation coefficients (ICC). All tests were two-sided, and *P* values < 0.05 were considered to indicate statistical significance.

## 3. Results

### 3.1. Baseline Characteristics

Table 1 compares baseline characteristics between the control group and the PCI group. There were no significant differences in age, sex, heart rate, body mass index, systolic blood pressure, diastolic blood pressure, and coronary heart disease-related risk factors between the control group and PCI group (*P* > 0.05).

### 3.2. Conventional Echocardiographic Variable

Table 2 manifests the conventional echocardiographic parameters between the two groups. Compared with the control group, LAD increased 1 day before surgery and 1 month after surgery, while LVIDd and LVIDs increased only 1 day before surgery; LVEF decreased 1 day before surgery and 1 month after surgery; the difference was statistically significant (*P* < 0.05); LVIDd decreased 1 month after surgery compared with 1 day before surgery; the difference was statistically significant (*P* < 0.05). There was no statistical difference in *E*/*e*′ between the PCI group and control group 1 day before surgery and 1 month after surgery (*P* > 0.05).

### 3.3. GLS and MW Parameters

Table 3 demonstrates the GLS and MW parameters between the two groups. Compared with the control group, the absolute value of GLS, GWI, GCW, and GWE in the PCI group decreased 1 day before surgery and 1 month after surgery, while GWW increased; the differences were statistically significant (*P* < 0.05). Compared with 1 day before surgery, the absolute value of GLS, GWI, and GCW increased 1 month after surgery; the differences were statistically significant. GWW and GWE were not statistically significant.

### 3.4. Correlation Analysis between Left Ventricular MW Parameters and GLS

There was a good correlation between MW parameters and GLS. GWI, GCW, and GWE were negatively correlated with GLS (*r* = −0.57, -0.53, and -0.61, all *P* < 0.05); GWW was positively correlated with GLS (*r* = 0.41, *P* < 0.05).

### 3.5. Reproducibility Test

The results indicate good repeatability of intraobserver and interobserver analysis results. The intraclass correlation coefficients for repeated measurements by the same observer (intraobserver agreement) were excellent for GWI (0.912) and GCW (0.887) and good for GWW (0.935) and GWE (0.932). The intraclass correlation coefficients for measurements between two different observers (interobserver agreement) were also excellent for GWI (0.940) and GCW (0.927) and good for GWW (0.863) and GWE (0.959) (all *P* < 0.001, see Table 4).

## 4. Discussion

PCI is a conventional invasive treatment for patients with NSTE-ACS, and early intervention can effectively reduce the occurrence of myocardial infarction [7], possibly lower the mortality of high-risk patients [8], and improve the prognosis of patients. Accurate assessment of the recovery of myocardial function after PCI is extremely important in these patients for clinical decision making and prognosis evaluation. Echocardiography has always been the preferred method to evaluate left ventricular systolic function, because of its noninvasive, economical, and simple advantages.

In recent years, a variety of new echocardiographic technology have been proved to be applicable to the evaluation of changes in myocardial function after PCI [9–12]. The evaluation of left ventricular systolic function is very important in cardiac diseases. LVEF is still the most commonly used parameter, but it is subjectively dependent. At the same time, myocardial motion is often affected by the pull of surrounding tissues. Therefore, the reproducibility of ejection fraction is poor, which reduces the accuracy of clinical application. STE can be used to quantitatively analyze left ventricular systolic function by tracking myocardial echo spots from the perspective of myocardial mechanics. STE has good repeatability, but there is still the effect of afterload dependency. Previous studies have shown that the increase of afterload will reduce the strain value, leading to the misunderstanding of the true systolic function of the left ventricle and the wrong conclusion of reduced myocardial function [2, 13], which underestimates the myocardial systolic function of patients. PSL is a new ultrasonic technology based on 2D-STE. Meanwhile, left ventricular pressure and strain are included in the study and analysis to overcome the influence of afterload to a certain extent [14]. PSL was used to quantitatively evaluate left ventricular myocardial work to observe changes in myocardial function after PCI, and the main parameters included myocardial work index, constructive work, wasted work, and work efficiency [15]. The analysis of global and regional myocardial work in patients with ST-segment elevation myocardial infarction before and after PCI has been discussed by scholars. It is believed that after primary PCI and optimal drug therapy, the regional myocardial work index of criminal vascular region before discharge is independently correlated with the early adverse left ventricular remodeling [16], which can predict the left ventricular remodeling before discharge, timely adjust the treatment measures, improve the survival rate of patients after discharge, and reduce the hospitalization rate. Other studies have shown that PSL can be used as a diagnostic tool for NSTE-ACS patients without obvious segmental ventricular wall motion abnormalities and normal LVEF, and it is believed that GWE can effectively predict severe coronary stenosis in NSTE-ACS patients, and its predictive value is superior to GLS and GWI [17–19]. It can be seen that PSL can not only predict the early remodeling of acute myocardial infarction but also identify patients with myocardial dysfunction and normal myocardial dysfunction shown by conventional echocardiography, improving the diagnostic rate of NSTE-ACS patients and providing a basis for accurate evaluation of myocardial function before clinical PCI.

There were no significant changes in general clinical data in this study. Conventional echocardiographic parameters, including LAD, LVIDd, LVIDs, and LVEF, were statistically significant compared with the control group one day before surgery, indicating that the left ventricular structure and function of NSTE-ACS patients were damaged, the diameter of the left ventricle was changed, and the left ventricular function was decreased to some extent. In the PCI group, LVIDd recovered 1 month after surgery, but LAD, LVIDs, and LVEF showed no significant difference from 1 day before surgery, indicating that myocardial function was not significantly improved 1 month after PCI. There was no statistically significant difference in *E*/*e*′ between patients before and after PCI, indicating that there was no significant change in left ventricular diastolic function. However, the evidence that *E*/*e*′ alone represented left ventricular diastolic function was insufficient. Changes in left ventricular diastolic function in patients with non-ST-segment elevation acute coronary syndrome require more studies and parameters.

Myocardial ischemia and hypoxia after coronary artery stenosis lead to myocardial dysfunction. Myocardial cell can be divided into stunned myocardium, hibernating myocardium, and scar myocardium (i.e., nonviable myocardium) due to different times of ischemia and hypoxia of myocardial cells. Stunned myocardium and hibernating myocardium are also known as viable myocardium. Myocardial damage is reversible, and it can be recovered within a certain amount of time after the narrowing is lifted in time. The prognosis of patients with myocardial injury is associated with survival myocardium number obviously, and the more the viable myocardium, the better the cardiac function recovery [20]. At the same time, some studies have shown that the existence of a certain amount of viable myocardium in the blood supply area of criminal blood vessels is the prerequisite for revascularization therapy to improve the prognosis [21]. In this study, the absolute value of GLS, GWI, GCW, and GWE was decreased and GWW was increased in the PCI group 1 day before surgery and 1 month after surgery (Figure 1), manifesting that the myocardial work of NSTE-ACS patients was reduced and left ventricular myocardial function was impaired. The absolute value of GLS, GWI, and GCW increased 1 month after surgery compared with that before surgery, while conventional echocardiographic parameters did not change significantly at this time, showing that the ability of left ventricular myocardial deformation in NSTE-ACS patients after PCI had been increased, the global myocardial work and the required useful work had been increased, and the left ventricular systolic function had been significantly improved. Previous studies have found that GLS can quantitatively evaluate the recovery of global and myocardial function of the left ventricle in patients with CHD after revascularization in an early and accurate way [22, 23]. However, GLS can only evaluate the deformation capacity of the left ventricle, which is not only affected by load conditions but also cannot reflect the oxygen consumption of the myocardium [24]. Russell et al. [14, 25] have confirmed that the noninvasive left ventricular PSL was significantly correlated with the invasively measured left ventricular PSL. Because the pressure-strain area loop reflected the metabolic demand and oxygen consumption of the myocardium, MW indirectly reflected the myocardial energy metabolism. A number of studies have demonstrated that PSL can effectively detect a variety of cardiovascular diseases and left ventricular dysfunction involving cardiac diseases [3, 26–28]. This study found that PSL can effectively assess the prognosis of patients with PCI at an early stage. Studies have shown that myocardial work can effectively evaluate the effect of cardiac resynchronization therapy (CRT) [29] and can be also used as a reliable complementary tool to guide the selection of patients with CRT in clinic [30]. In this study, GLS and myocardial work parameters still decreased 1 month after surgery compared with the control group, indicating that myocardial systolic function did not return to the normal level at this time. Therefore, it is necessary to further follow up these patients after PCI to observe their long-term prognosis after PCI. The correlation between MW parameters and GLS is good. Therefore, PSL will hopefully become a new method for the evaluation of subclinical myocardial dysfunction, with considerable development prospects.

## 5. Limitations

The limitations of this study are as follows: (1) this study was a single-center study with a small sample size, so it is necessary to further enlarge the sample size to improve the accuracy of the study; (2) the follow-up time was too short, and the long-term efficacy after PCI was not clear; (3) the left ventricular pressure used in PSL was replaced by brachial artery systolic pressure, which could not accurately evaluate patients with severe aortic stenosis and left ventricular outflow tract obstruction; (4) only *E*/*e*′ was included in the evaluation of diastolic function, and multiple parameters were not combined to explore; (5) the regional myocardial function was not studied and needs further investigation; and (6) we mentioned the results of coronary angiography briefly, but the clinical medication of each patient was not included in the study.

## 6. Conclusion

In conclusion, the myocardial function of NSTE-ACS patients is impaired to varying degrees. The PSL technology can quantitatively evaluate the global systolic function of the left ventricle at an early stage, providing a new noninvasive method for the prognosis evaluation of patients after PCI, and has very important guiding significance for further clinical treatment.

## Figures and Tables

**Figure 1:** Pressure-strain loop and 17 segments of the left ventricular myocardium for bull's eye: (a) left ventricular PSL in a normal subject; (b) left ventricular PSL of a patient in the PCI group 1 day before surgery; (c) left ventricular PSL of the same patient in the PCI group 1 month after surgery.

**Table 1:** Patient characteristics of the control and PCI group.

Patient characteristics	Control group (*n* = 30)	PCI group (*n* = 33)	*t* or *χ* value	*P* value
Age (years)	58.50 ± 6.70	62.09 ± 9.16	-1.761	0.083
Male (%)	20 (66.7)	25 (75.8)	0.636	0.425
BMI (kg/m^2^)	23.81 ± 2.47	24.47 ± 2.69	-1.014	0.315
Heart rate (bpm)	70.07 ± 8.29	67.18 ± 7.27	1.472	0.146
Systolic BP (mmHg)	123.13 ± 10.34	128.33 ± 12.92	-1.752	0.085
Diastolic BP (mmHg)	75.67 ± 8.67	74.21 ± 9.28	0.641	0.524
Diabetes mellitus (*n*)	6 (20.0)	12 (36.4)	2.062	0.151
Dyslipidemia (*n*)	9 (30.0)	13 (39.4)	0.610	0.435
Smoking (*n*)	6 (20.0)	10 (30.3)	0.880	0.348

1 mmHg = 0.133 kPa; BMI: body mass index.

**Table 2:** Conventional echocardiographic analysis of control patients versus PCI patients.

	Subjects, *n*	LAD (mm)	LVIDd (mm)	LVIDs (mm)	*E*/*e*′	LVEF (%)
Control group	30	35.27 ± 3.35	47.13 ± 3.53	29.20 ± 3.21	9.63 ± 2.43	64.27 ± 2.15
PCI group	33					
1 day before surgery		39.15 ± 3.95^a^	51.03 ± 3.43^a^	30.91 ± 3.43^a^	11.36 ± 3.68	59.06 ± 2.62^a^
1 month after surgery		38.21 ± 3.40^a^	48.58 ± 2.94^b^	29.91 ± 2.99	11.09 ± 3.50	59.82 ± 2.83^a^
*F*/*H* value		9.922	11.294	2.254	4.189	37.319
*P* value		*P* < 0.01	*P* < 0.01	0.111	0.123	*P* < 0.01

Compared with the control group, ^a^*P* < 0.05; compared with PCI group 1 day before surgery, ^b^*P* < 0.05.

**Table 3:** GLS and MW analysis of control patients versus PCI patients.

	Subjects, *n*	GLS (%)	GWI (mmHg%)	GCW (mmHg%)	GWW (mmHg%)	GWE (%)
Control group	30	−21.60 ± 1.27	2038.83 ± 165.54	2379.73 ± 204.72	79.33 ± 32.18	96.23 ± 1.28
PCI group	33					
1 day before surgery		−17.74 ± 1.65^a^	1719.88 ± 308.49^a^	2048.12 ± 365.43^a^	153.67 ± 72.07^a^	91.88 ± 2.82^a^
1 month after surgery		-18.70 ± 1.46^ab^	1847.30 ± 248.03^ab^	2190.03 ± 264.29^ab^	138.06 ± 58.46^a^	93.39 ± 2.16^a^
*F*/*H* value		57.567	12.902	10.254	26.334	41.137
*P* value		*P* < 0.01	*P* < 0.01	*P* < 0.01	*P* < 0.01	*P* < 0.01

Compared with the control group, ^a^*P* < 0.05; compared with the PCI group 1 day before surgery, ^b^*P* < 0.05.

**Table 4:** Reproducibility test of MW parameters.

Parameters	Interobserver		Intraobserver	
	ICC	95% CI	ICC	95% CI
GWI	0.912	0.688~0.977	0.940	0.762~0.985
GCW	0.887	0.607~0.971	0.927	0.749~0.981
GWW	0.935	0.674~0.965	0.863	0.517~0.965
GWE	0.932	0.719~0.983	0.959	0.853~0.989

CI: confidence interval.

## Data Availability

All the data associated with this study can be accessed by requesting to the corresponding author.

## Abbreviations

PSL: Pressure-strain loop
NSTE-ACS: Non-ST-segment elevation acute coronary syndrome
PCI: Percutaneous coronary intervention
LVEF: Left ventricular ejection fraction
STE: Speckle tracking echocardiography
GLS: Global longitudinal strain
MW: Myocardial work
GWI: Global work index
GCW: Global constructive work
GWW: Global wasted work
GWE: Global work efficiency
BMI: Body mass index
LAD: Left atrium diameter
LVIDd: Left ventricular internal diameter end diastole
LVIDs: Left ventricular internal diameter end systole.
